# The Characteristics and Paths of the Dissemination of Intangible Cultural Heritage in the Form of Animation in the New Media Environment

This article has been retracted.

**DOI:** 10.1155/2022/7857816

**Published:** 2022-07-30

**Authors:** Jie Luo

**Affiliations:** School of Gannan Normal University, Ganzhou 341000, China

## Abstract

In recent years, the state and even the society pay more and more attention to the protection of the intangible cultural heritage. How to effectively protect and inherit the intangible cultural heritage is the main work at present. Based on the role and influence of animation in the protection of intangible cultural heritage, this paper systematically discusses the promotion role of animation in the inheritance and dissemination of intangible cultural heritage. First, the role of animation communication in the protection of intangible cultural heritage. Finally, this paper takes the combination of intangible cultural heritage culture and animation as an example to discuss and design the combination of intangible cultural heritage protection animation and specific cases. This paper regards animation as a cultural medium, which is of great significance to the effective protection, dissemination, and inheritance of the national intangible cultural heritage.

## 1. Introduction

The heritage of nontraditional culture allows people to appreciate the greatness of human history on the one hand and to realize the importance of environmental energy efficiency on the other. In the process of learning about nonheritage culture, we can learn a lot about traditional handicrafts and nonindustrial forms of life and production. Web animation is a more visual, easier to understand, and more widespread way of presenting nonheritage culture. The use of web animation can raise awareness among the younger generation about the heritage and the need to save energy in the environment.

Because we do not have enough understanding of intangible cultural heritage, a lot of intangible cultural heritage is gradually dying; in terms of drama, for example, before the reform and opening up, China had more than 300 local dramas, Influenced by trendy culture, there are only a few dozen varieties left today.

The protection of intangible cultural heritage has gradually been paid attention to in recent years. This is because the original soil of the preindustrial society as intangible cultural heritage has gradually disappeared and the global integration of modern society has brought huge impact on traditional social forms. It is difficult to survive by relying on its own internal cultural system, and we must rely on external forces to protect it [1]. As a kind of spiritual inheritance, the protection of intangible cultural heritage is more about maintaining the continuation of its vitality, which is a long-term work based on the present and looking forward to the future. Therefore, the investigation, recording, preservation and subsequent dissemination, promotion, inheritance, and revitalization of intangible cultural heritage are what the protection of intangible cultural heritage in contemporary society must do [2].

## 2. Innovation in the Way of Dissemination of Intangible Cultural Heritage

As mentioned above, the dissemination of intangible cultural heritage is what a contemporary society must do in the protection of intangible cultural heritage. Therefore, we need to think about how to spread and through what way. Four different novel modes of propagation are listed in Figure 1.

### 2.1. Establishment of a Reconnection with Contemporary Life

The vitality of intangible cultural heritage lies in the close connection with people's lives. Therefore, it is far from enough to rely only on individual inheritors to inherit within a specific cultural protection circle, which makes the inheritance isolated and closed and has almost no intersection with the life of the general public. The barrier of protection will eventually die out [3]. Intangible cultural heritage used to be an important part of our lives, so although times have changed and cultures have migrated, this way of completely detaching from life cannot gain strong vitality. Therefore, intangible cultural heritage should be flushed with modern life to establish a connection. Although it cannot return to the core position of people's production and life, it can return to people's life as a part of cultural composition [4]. For example, due to the broadcast of the cartoon “Lucky Star,” the number of visits to the Chu Palace Shrine has increased year by year, as shown in Figure 2.

### 2.2. Reconstruction of Intangible Cultural Heritage Functions

The main function of intangible cultural heritage is to spread ethnic culture and increase cultural confidence. For example, paper-cutting can be used as decoration and tie-dyeing technology can be used as clothing dyeing. Due to the development and progress of science and technology, people's production and lifestyle have been completely different from the original, which has led to the gradual disappearance of the original use function of many intangible cultural heritages, which is one of the main reasons for the difficulty of inheriting intangible cultural heritage. Whether the functionality can be re-realized is an important basis for considering whether the intangible cultural heritage can continue to develop and survive [5]. Therefore, in modern society, it is necessary to rebuild the functionality of intangible cultural heritage with the help of new conditions and technologies, so that it can continue to be passed on proudly.

### 2.3. Recultivation of Cultural Identity

If a culture wants to have a strong vitality, the identity of the people as a communication medium is very important. A good cultural atmosphere can provide fertile soil for the inheritance of intangible cultural heritage. People recognize this culture, understand its cultural value and connotation, and realize the importance of protecting intangible cultural heritage, so as to build a good atmosphere for intangible cultural heritage protection [6]. It also makes the people themselves consciously realize their important role in the inheritance of intangible cultural heritage, so that human beings can spontaneously protect and inherit the intangible cultural heritage.

### 2.4. Changes in the Way of Inheritance

For the inheritance of intangible cultural heritage in the contemporary cultural context, in addition to the reconnection with people's lives, the reconstruction of functions, and the recultivation of cultural pride mentioned above, it is also necessary to take measures to improve the spontaneous inheritance of intangible cultural heritage [7]. Borrowing external forces to promote the inheritance of intangible cultural heritage, the search for new media bears the brunt. As a sunrise industry, animation has a natural property of integrating with modern fast-paced cultural dissemination. As a pioneer representative of visual culture and an important part of contemporary cultural industry, animation is very suitable for the inheritance of intangible cultural heritage as a new media [8]. The communication mode of the animation industry in the intangible cultural heritage is shown in Figure 3.

## 3. The Feasibility Analysis of the Communication Characteristics and Communication Paths of the Intangible Cultural Heritage Animation in the New Media Era

### 3.1. The Communication Characteristics of the Intangible Cultural Heritage Animation in the New Media Era

In the process of protecting intangible cultural heritage, it is particularly important to preserve relevant data materials. The protection of folk art is the core part of the process of intangible cultural heritage protection. The inheritance and development of folk art are essentially the inheritance and development of the national spirit and culture. The study of historical and cultural heritage needs to reflect the textual nature of history. With the characteristics of diversification and life, folk art has played a unique cultural function in modern civilization, which is very important to strengthen national unity and enhance people's sense of collective identity. From a historical point of view, folk art is an important guarantee for maintaining the diversity of human culture and the foundation for the healthy development of the cultural ecosystem [9]. At the same time, the relevant personnel also encountered some difficulties in the process of protection. The dissemination of intangible cultural heritage is a dynamic transmission with human beings as the carrier, which is transmitted by oral transmission [10]. This inheritance method is very dependent on the inheritors, and it is very easy to cause the decay or loss of cultural connotations in the process of dissemination. With the continuous advancement of globalization and digitalization, the emergence of new forms of media has brought a certain impact on the dissemination of intangible cultural heritage. The traditional dissemination and promotion of intangible cultural heritage mainly relies on oral, written, picture, and other forms; if the original mode of communication is continued without innovation, intangible cultural heritage may face the embarrassing situation of being snubbed. We have to think about new channels and ways of disseminating intangible cultural heritage. In the face of the transition between tradition and modernity, intangible cultural heritage culture needs to be combined with the form of animation, which plays an important role [11]. Animation in the protection and dissemination of intangible cultural heritage mainly can be carried out through the three latitudes as shown in Figure 4.

#### 3.1.1. Animation Works Can Better Protect and Express the Essence of Folk Art

At present, our country mainly protects and develops folk art by applying folk art forms as intangible cultural heritage projects, systematically sorting out folk art, selecting inheritors and cultivating them, and rationally developing projects with economic value. In the process of protecting and inheriting intangible cultural heritage, the protection concept of relevant personnel is relatively old and the technology is single. They only preserve and record the intangible cultural heritage by means of photography, recording, or physical collection, and these preservation methods may change over time. The passage of time leads to the distortion of some information. As a new medium, animation works preserve the essence of folk art in digital form, which can be a useful supplement to the traditional record and preservation work [12].

#### 3.1.2. Animation Works Can Play a Good Role in Inheritance

The audience of animation products is very wide, and the vividness of animation has a strong appeal to young people. In recent years, with the continuous development of the animation industry, a large-scale group of animation enthusiasts has formed among the youth groups and even the adult groups. These fans maintain high enthusiasm for domestic animation works, such as “Journey to the West: The Return of the Great Sage” and “Big Fish and Begonia” in recent years, which have caused quite a stir. Animation works with excellent traditional cultural themes can express excellent traditional art, promote excellent traditional culture, activate the national enthusiasm and cultural enthusiasm of the younger generation, enhance their sense of national pride and identity, enhance the interest of young people in traditional culture and art, and make folk culture and art get a better inheritance [13]. For example, the soul of the Japanese anime directly affects the number of Japanese participants in Go, as shown in Figure 5.

#### 3.1.3. Animation Is Conducive to the Sound Development of the National Cultural Industry

The animation industry is a cultural and creative industry, and animation creators need to have advanced and avant-garde creative concepts and skills. However, looking at the excellent animation works of different countries, distinctive national characteristics are the basis for their long-term development. Only animation works with unique national character can have product differentiation and improve their competitiveness in the international cultural market. Animation works have a strong cross-cultural communication ability. In order to exert this ability, animation creators need to find a basis from the excellent cultural and artistic traditions of their own nation. Today, with the deepening of the process of globalization, the trend of interpenetration and integration of cultures among different civilizations and nations is increasing. Under this background, in order to achieve good development of domestic animation, it needs to be effectively integrated with intangible cultural heritage, which is also a necessary means of disseminating and protecting national intangible cultural heritage and is of great significance for ensuring the safety of national culture [14].

### 3.2. The Feasibility of Nongenetic Inheritance Using Animation as a Medium

The subject matter of animation can be described as all-encompassing, from sci-fi adventure to campus romance to sports humor. Therefore, the dissemination of intangible cultural heritage by animation is also diversified.

#### 3.2.1. The Breadth of the Creative Subject Matter

The wide range of performance themes just proves the strong integration ability and expressive power of animation to culture. The wide range of themes is the fertile soil for animation to grow, showing us the excellent culture of the genre and conveying the connection between nature and human society [15].

#### 3.2.2. Diversity of Performance Materials

The essence of animation is “the art of motion.” As long as it is the material that can be applied to animation shooting and form motion, it can be used as the object of animation performance. The use of different materials can bring more expressiveness and tension to the expressiveness of animation. With the advent of the digital age in today's society, optical virtual animation based on computer technology uses computer three-dimensional virtual animation to complete the corresponding three-dimensional model construction. It can realistically and directly build an actionable visual virtual reality scene for the user, completely separated from the performance of physical materials, bringing new creative vitality to the performance of animation.

#### 3.2.3. Compatibility of Artistic Application

As a comprehensive art, the compatibility of animation with other disciplines such as literature, music, sculpture, and dance is unmatched by other art forms. The absorption and transformation of excellent literary works in animation creation, the use of excellent musical works in sound, and the reference to sculpture and dance in art design all reflect the compatibility and breadth of an art form [16].

#### 3.2.4. Diversity of Forms of Communication

The form of communication of animation has changed from the early paper media such as newspapers, magazines, and comics, to the medium of television as the main communication medium, to the network as the main communication medium in contemporary society. No matter which period the animation media has a strong audience base, its popularity is unmatched by other art forms. From a macro point of view, the communication forms of animation cover all aspects from traditional media to new media, and an open and flexible communication system has been spontaneously formed [17].

#### 3.2.5. Rich Intangible Cultural Heritage Resources Provide Materials for Animation

Our country's intangible cultural heritage resources are rich in different forms. As of December 31, 2019, according to relevant statistics, there are 3,145 intangible cultural heritage items in my country, which are divided into folk literature, traditional music, traditional dance, traditional drama, folk art, traditional sports, entertainment and acrobatics, traditional art, traditional Skills, traditional medicine, and folk customs comprising 10 categories. These various types of intangible cultural heritage have high artistic and cultural value and continue to provide rich materials for animation creation in our country, as shown in Table 1.

#### 3.2.6. The Combination of Intangible Cultural Heritage Culture and Animation Has a Long History

With a long history of combining intangible cultural heritage culture with animation, Table 2 integrates relevant specific information.

### 3.3. The Dissemination Path of Animation of Intangible Cultural Heritage in the Era of New

#### 3.3.1. Strengthening Psychothematic Analysis

Although the dissemination of intangible cultural heritage by means of animation will weaken the charm of intangible cultural heritage, in order to make it spread, it is also necessary to spread intangible cultural heritage by means of animation. The dissemination of intangible cultural heritage by means of animation is actually a second creation of intangible cultural heritage. China's intangible cultural heritage contains the outstanding wisdom and cognitive experience accumulated by the ancestors of the Chinese nation for generations, as well as the spiritual connotation of traditional culture such as continuous self-improvement and virtue for generations, providing strong cohesion and inexhaustible creativity for the Chinese people. As a creator, we must be able to grasp the theme spirit of intangible cultural heritage as much as possible and be able to grasp its core connotation. Based on this, we carry out animation processing and try to display the essence of intangible cultural heritage, so that the dissemination of intangible cultural heritage has practical value. Specifically, if the creation is too heavy, it is necessary to seriously study the ecological structure of the intangible cultural heritage, the human situation, and the philosophy of life. Its spiritual qualities are effectively disseminated. Animation creators must be able to study nonmaterial cultural works in depth, to deeply grasp their connotations, and to grasp their spiritual qualities. In line with the esthetic needs of modern people, it can also show the spiritual quality of intangible cultural heritage as much as possible. In this way, intangible cultural heritage can be disseminated so that people can deeply appreciate the spiritual charm and cultural charm of intangible cultural heritage through phenomena. This kind of dissemination has real value.

#### 3.3.2. Scientifically Building Image Pedigree

In the era of new media, in order to realize the animation dissemination of intangible cultural heritage, it is necessary to be able to scientifically construct the image genealogy, that is, animated films must continuously enter new content and create an innovative cultural environment, as the most novel cultural form, which is the basic guarantee for its effective dissemination, as shown in Table 3. To scientifically build an image pedigree, we need to be able to analyze the characteristics of intangible cultural heritage, and combine the advantages of new media to create an animation image brand that belongs to intangible cultural heritage. This animation image brand can effectively enhance the influence of intangible cultural heritage and enhance the market competitiveness of animation products, so that intangible cultural heritage can be effectively disseminated.

#### 3.3.3. Analysis of Esthetic Appeals

The animation design of intangible cultural heritage needs to be able to analyze the aesthetic appeal of modern people. As a kind of traditional culture, intangible cultural heritage is produced in a specific historical period, and its esthetic expression cannot well meet the aesthetic needs of modern people, which is also an important reason for the difficulty of dissemination of intangible cultural heritage. To carry out animation design and dissemination of intangible cultural heritage through animation, it is necessary to be able to carefully analyze the esthetic appeals of modern people and to be able to effectively design the manifestations of intangible cultural heritage based on the esthetics of modern people. Through animation design and creation, intangible cultural heritage can be welcomed by the audience. In the process of creation, creators should be able to deeply study the spiritual connotation of intangible cultural heritage, and should be able to design artistic situations that are compatible with classic works. It is closer to the esthetic appeal of modern people. In this way, intangible cultural heritage can be effectively disseminated by means of animation, and its sustainable development and creative development can be guaranteed.

Chinese ink painting is a traditional element in Chinese animation. In the expression of situations and the creation of artistic conception, the artistic elements of ink painting are widely used and have strong performance advantages. In the animation design, many works are designed with the artistic element of ink painting which renders an atmosphere and conveys a national spirit. This design also meets the aesthetic needs of modern people. Therefore, this ink painting anime design is very popular.

#### 3.3.4. Creation of Animation Works with the Theme of Intangible Cultural Heritage

In order to solve the problem of the marginalization of intangible cultural heritage elements in animation works, my country should vigorously support the creation of animation works with intangible cultural heritage as the theme at this stage. In 2004, our country's CCTV Variety Channel launched an animation column with the theme of intangible cultural heritage, “Happy Station,” which performed intangible cultural heritage projects such as Chinese classic humorous comic dialogue, storytelling, and sketches in the form of animation. After the program was broadcast, it not only received unanimous praise from middle-aged and elderly audiences who love traditional folk art but also had a warm response among young people, which had a positive impact on the inheritance of traditional folk art. Intangible cultural heritage has not received much attention among contemporary youth groups, and inheritance is faced with the dilemma of no successor. Under this situation, the cultural connotation of intangible cultural heritage should be fully explored, and different animation expressions should be adopted to display intangible cultural heritage under the premise of grasping the characteristics of different types of intangible cultural heritage items as shown in Table 4.

It is worth noting that when creating art forms, the authenticity of intangible cultural heritage should not be neglected, and the relationship between entertainment and seriousness should be well handled, so as to stimulate young people's interest in intangible cultural heritage and encourage them to devote themselves to the development of intangible cultural heritage inheritance.

#### 3.3.5. Building a Professional Intangible Cultural Heritage Animation Creation Team

The animation of intangible cultural heritage is a complex task. The final effect of the work is not only reflected in the visual perception but also depends on the content of the work, which requires the joint participation of talents from all parties. Excellent animation designers can ensure the artistry of the work, and the participation of intangible talents ensures the authenticity and accuracy of the work. The lack of any talent will lead to the failure of the work. Therefore, our country should vigorously cultivate animation creative talents with innovative consciousness and production ability, and at the same time, it should also attract more intangible cultural heritage talents to participate in animation creation and build a professional intangible cultural heritage animation creation team.

#### 3.3.6. Increasing the Popularization of Intangible Cultural Heritage Elements in Works

There are many works involving intangible cultural heritage elements in domestic animation, but there are very few related introductions to the intangible cultural heritage elements. As a result, some audiences are attracted by the intangible cultural heritage elements in the works and want to know more about them, but they cannot find more relevant information. The animation production team can mark the intangible cultural heritage elements borrowed from the work at the end of the subtitle, so that the audience has a general direction and can check the relevant information on their own. At the same time, the production team can also use social media such as Weibo to publish popular science articles or related introduction videos of the intangible cultural heritage projects involved in the work, so as to increase the public's understanding and familiarity with intangible cultural heritage and promote the inheritance of intangible cultural heritage [18].

In a word, intangible cultural heritage originated in a specific historical period and a specific historical culture. As an important carrier of national culture and national spirit, it plays a positive role in the dissemination of traditional Chinese civilization. Therefore, strengthening the inheritance and protection of intangible culture is very important. In the new era, people's life rhythm has been accelerating, and esthetic needs have also undergone great changes [19]. People's attention to intangible cultural heritage has gradually declined, and it has become more difficult to spread intangible cultural heritage. In this case, in order to realize the inheritance and dissemination of intangible cultural heritage, it is necessary to carry out animation design of intangible cultural heritage based on the needs of the development of the new media era and to carry out intangible cultural heritage dissemination in the way of animation. In this way, the traditional art elements are recreated to meet the esthetic needs of modern people. Only in this way can we effectively create a unique brand of intangible cultural heritage and promote the innovative development of intangible cultural heritage [20].

## 4. Case Analysis of the Inheritance and Dissemination of Intangible Cultural Heritage Animation Industrialization

### 4.1. Inheritance and Dissemination of Animation Industrialization of Intangible Cultural Heritage—Taking Yinxu of Anyang as an Example

The animation industrialization of intangible cultural heritage refers to the combination of intangible cultural heritage and the animation industry, and through the integration of resources, the intangible cultural heritage becomes a cultural resource and a source of creativity for animation creation, so that it can participate in animation creation, derivative development and industry in operation. We will take Yin Ruins in Anyang, Henan Province as an example to discuss specific and implementable cases of intangible cultural heritage animation and animation industrialization, to highlight the feasibility of intangible cultural heritage with animation as the way of communication.

#### 4.1.1. Animation Creation: The Transformation of Intangible Cultural Heritage to Animation Symbols

The original obscure oracle bone script was transformed into animation language and expressed in the form of modern animation to establish its connection with the animation industry. Creativity is the source of power for the cultural industry. It runs through the entire industry, and cultural products produced with creativity as the driving force are the most intuitive visual manifestations. Taking intangible cultural heritage as the source of cultural creativity refers to taking intangible cultural heritage elements as the object of animation creation and using intangible cultural heritage as the content of animation performance, so that intangible cultural heritage can be integrated into the animation industry chain.

#### 4.1.2. Cultural Derivatives: Diversified Dissemination of Intangible Cultural Heritage

In the context of contemporary cross-media communication, animation visual derivatives are an important part of animation products and are visual cultural products that use existing animation symbols to develop other types of media and functions. The development of animation visual derivatives provides more communication channels for animation symbols, and at the same time, enriches their forms of expression and presentation. Animation, games, and cultural and creative products are all available channels. Oracle bone inscriptions and modern Chinese have a natural inextricable relationship which is very suitable for the development of early childhood education products of Chinese characters for children and can also be developed in the form of the most popular modern mobile phone app. The shape is transformed into an animation image, and the origin of modern Chinese characters is linked to the origin of oracle bone inscriptions.

#### 4.1.3. Physical Derivatives: New Functional Construction of Intangible Cultural Heritage

The development of animation physical derivatives refers to the development and sales of physical products of related animation symbols and contents through the grant of animation copyrights. The development of animation physical derivatives is the most direct means of adding value to animation symbols, and it is also an important link for the animation industry to promote the related manufacturing economy. The “complex” caused by the cartoon symbols condensed in the physical products is the biggest attraction for consumers. At the same time, in the process of physical development, intangible cultural heritage has unconsciously formed new functions. In the contemporary era of advocating individuality and trends, young people are very fond of individual culture. The shape of oracle bone inscriptions is a very individual cultural symbol. Wearing it directly as a kind of jewelry not only satisfies young people's pursuit of individuality but also using people as a communication medium has also played a very good role in the spread of Oracle. This is actually a new construction of the functionality of the intangible cultural heritage, which migrates the original recording and communication function of oracle bone inscriptions into the modern cultural aesthetic function, satisfies the pursuit of individual culture, and activates the new function of intangible cultural heritage.

#### 4.1.4. Combining with Contemporary Tourism

Combining animation with intangible cultural heritage and tourism refers to a series of tourism products formed by combining animation resources with local tourism resources. There are two modes for packaging tourism by symbolizing intangible cultural heritage animation. First, we symbolize intangible cultural heritage items with animation to enhance their appeal to the audience. We can carry out animation packaging for the image of the explainer, for example, let him dress as the image of an ancient cartoon character, which can make the audience more immersive than the modern professional dress. Second, we develop cartoon images to create highly recognizable symbols for intangible cultural heritage tourism projects.

### 4.2. Inheritance and Dissemination of Animation Industrialization of Intangible Cultural Heritage—Taking the Resource River Lantern Festival as an Example

We will take the Resource River Lantern Festival as an example to discuss the specific and implementable cases of intangible cultural heritage animation dissemination.

#### 4.2.1. Improving the Quality of Intangible Cultural Heritage Content Dissemination

With the rapid development of new media, their relevant content and form are very critical. Therefore, it is necessary to combine the development of the Internet to create more high-quality works. Through new media, designers can use new media technology to create animation materials, and can also obtain more materials through network channels. In the design of the works, through the use of nonperspective composition, multiple viewpoints in ancient Chinese painting, and ethnic color elements, the boring traditional text introduction to the River Lantern Festival has been transformed into novel and visual animation works. At the same time, dynamic illustrations are used to make the picture more rich and interesting. Finally, you can disassemble the elements of the River Lantern Festival, make stamps, tapes, bookmarks, posters, and other products, play with creativity, design derivatives, outline static and dynamic cultural surroundings, and make it more widely used.

#### 4.2.2. Making Full Use of New Media Forms to Innovate Network Communication Channels

At present, the River Lantern Festival, which is an intangible cultural heritage, is mainly concentrated on news websites. From this point of view, we should make reasonable use of various channels and forms of existing network communication, so as to cover more netizens more effectively and achieve the effect of expanding communication. In terms of visual communication, H5 video can be produced. The meaning of river lanterns, worshiping gods and ancestors, birds and beasts, flowers, birds, fish and insects, Baolian blessings, scenic spots, festivals and activities and special neighborhoods, special food, and special residential properties will be introduced in the “interactive videos” is presented one by one, so that the culture of the River Lantern Festival can be presented to the public in the form of information visualization. It is also possible to create a digital resource He Lantern Festival special website, fully consider the acceptance habits of Internet users, and use a variety of symbolic media such as text, pictures, sound, and video.

#### 4.2.3. Using Social Network Media Skillfully for Dissemination

The emergence of new media has brought more convenient communication methods to the animation industry. Various websites, platforms, and apps for the animation industry emerge in an endless stream. Not only are there various types, but also the number of online users is on a linear upward trend, which greatly broadens the dissemination channels of animation. IMoreover, in addition to animation works, a series of animation derivatives can also be produced, which makes the development trend of animation works appear diversified. In addition, with the gradual popularization of the Internet and the continuous development and maturity of network technology, “interaction design” can also be used in the dissemination of animation works. In this context, we can use WeChat public account, Weibo, major self-media platforms, etc., with the help of the Internet, short videos, mobile phones, and other technologies to disseminate animation works that consumers love to hear and provide users with effective science resources for the River Lantern Festival.

## 5. Conclusion

This paper explores and studies the ways in which intangible cultural heritage can be disseminated and transmitted in the new media era. After demonstration, it was found that animation, as a medium and form, can be effectively combined with intangible cultural heritage and promote the inheritance and dissemination of contemporary intangible cultural heritage. By analyzing the survival dilemma of intangible cultural heritage due to the loss of its original function in the contemporary cultural context, this paper finds that the intervention of modern media can find a way out through mass communication and industrial inheritance. At the same time, it is proved that animation can integrate intangible cultural heritage elements into the industrial chain from three different dimensions of animation, and inherit and disseminate intangible cultural heritage through cultural products and tourism development. Finally, taking the combination of intangible cultural heritage and animation in many places as an example, it specifically pointed out how to transform intangible cultural heritage into animation form, and demonstrated its feasibility in the production of physical projects.

## Figures and Tables

**Figure 1:** Innovation in the way of dissemination of intangible cultural heritage.

**Figure 2:** Changes of the number of visits to the animation Lucky Star and the Chu Palace Shrine.

**Figure 3:** Industrialization mode of intangible cultural heritage animation.

**Figure 4:** Three dimensions of anime.

**Figure 5:** Population change chart of Go Soul and Japanese Go.

**Table 1:** Rich intangible cultural heritage resources provide materials for animation.

The Eight Immortals Crossing the Sea“, “The Story of Avanti“, “Da Yu's Control of the Flood“ and “White Snake: The Origin”	Based on Chinese folk tales
“Havoc in Heaven“ and “The Return of the Great Sage”	The soundtrack draws on traditional musical elements such as Peking Opera, Kunqu Opera, and Guangdong Cantonese Opera
“Fisher Boy“, “Gourd Brothers“ and “Monkey Fishing for the Moon”	The soundtrack are paper-cut animations based on traditional art creations
“Legend of Shaolin“ and “Go Boy”	Draw on traditional sports, entertainment and acrobatics intangible cultural heritage projects
“Herbal Family“ and “Ben Herbal Spirit”	Take traditional medicine as the theme
“Dao Xi“	Takes the inheritance of Hunan “Dong Brocade” as the main line

**Table 2:** The combination of intangible cultural heritage culture and animation history.

1940s	“Princess Iron Fan”	Paper cutting, puppets, fine brushwork, ink painting, shadow play, etc.

From the 1960s to the end of the 1980s	“The Proud General” and “Havoc in Heaven”	For example, the classic image of Monkey King in “Havoc in Heaven“, its facial design absorbs the elements of Peking Opera masks, and the costumes incorporate tiger skin skirts, drill hats and other elements commonly seen in operas, and use the form of folk prints to outline the character as a whole. In “Nezha Nao Hai“, the shape of the Dragon King is inspired by folk paper-cuts and New Year pictures. The music in these animation works is also played with traditional musical instruments such as drums, cymbals, and suonas, reflecting the strong characteristics of traditional drama.
	“Mud Flute”	
	“Little Tadpoles Looking for Mother”	
	“Nine Colored Deer”	
	“Landscape Love”	

After the 21st century	“The Legend of Panhu”	At the beginning of production, it is consciously combined with intangible cultural heritage, which is a great progress, which can break through the shackles of inherent communication forms and attract the interest of young people.
	“Cai Lifo, the Hero of Star Ants”	

**Table 3:** Scientifically constructed image pedigree.

In the dissemination of Chinese opera culture	Using animation expression to display traditional opera stories, designing the story situation through secondary creation, and enriching and perfecting relevant details, this animation product is more artistic, and the dissemination of Chinese opera in this way can make the audience feel Chinese opera has a more profound impression, so that the effective dissemination of Chinese opera art can be realized.

During the adaptation of the classic opera “The Legend of the White Snake”	During the animation adaptation process, the creators made a scientific construction of the image pedigree, and effectively displayed the surrounding scenery of the West Lake through delicate and elegant traditional ink brushwork, creating a fresh and elegant artistic atmosphere.
	In terms of character image design, the creators used exaggerated methods to display the character characteristics of the characters, which effectively enhanced the impact of the image. The appeal of the work enables the widespread dissemination of intangible cultural heritage

**Table 4:** Different ways of expressing intangible cultural heritage in animation.

Folk literature	This kind of intangible cultural heritage that is mainly narrative can show the storyline through the direct creation of cartoons.

Other types of intangible cultural heritage	This can use the existing well-known animation images to promote intangible cultural heritage or use 3D animation technology and VR technology to create a virtual animation scene, the audience can watch the intangible cultural heritage project up close and even participate in it.

## Data Availability

The labeled data set used to support the findings of this study is available from the author upon request.
